# Computational Intelligence Powered Experimental Test on Energy Consumption Characteristics of Cold-Water Phase-Change Energy Heat Pump System

**DOI:** 10.1155/2022/1941855

**Published:** 2022-09-06

**Authors:** Ronghua Wu, Hao Yu, Ying Xu

**Affiliations:** ^1^College of Mechanical and Electrical Engineering, Qingdao University, Qingdao 266071, Shandong, China; ^2^Qingdao Kechuang Blue New Energy Co., Ltd., Qingdao 266300, Shandong, China; ^3^Harbin University of Commerce, School of Energy and Architecture Engineering, Heilongjiang, Harbin 150028, China

## Abstract

In order to study the influence on the effective energy efficiency ratio, the energy consumption characteristics of a cold-water phase change heat pump system are discussed in this article. An experimental system of the cold-water phase-change energy heat pump system is designed and constructed, and then the deicing energy consumption and unit energy consumption of the heat pump system are analyzed by computational intelligence-powered methods. At last, the primary energy utilization ratio of the heat pump system is calculated. The results show that under the setting conditions, the deicing capacity of the heat pump system is about 0.135, the primary energy utilization ratio is about 1.145, and the COP (coefficient of performance) of the heat pump unit is between 2.8 and 3.2. Considering the system's deicing energy consumption, the effective COP of the unit is between 2.42 and 2.76, so from this point, this kind of heat pump system can be widely used in the future. In order to improve the effective COP of the unit, the processes of ice making and melting should be further optimized to reduce heat loss and power loss.

## 1. Introduction

Using cold-water phase-change energy heat pump technology for building, heating, and cooling has great economic and environmental benefits. Cold-water phase-change energy heat pump technology is a new technology that uses a phase-change heat exchanger to extract latent heat of phase-change in water for heating and cooling [1]. Under the same heating conditions, the cold-water phase-change energy heat pump technology theoretically needs only 1/16 of the water volume in the existing water source heat pump system, which expands the application scope of heat pump technology [2–5]. At present, some domestic scholars are studying a part of the research work on the cold-water phase-change energy heat pump system; most of them are focusing on the research and development of the system and the icing mechanism. In the aspect of energy consumption characteristics of the heat pump system, there are few studies domestic and abroad. However, the energy consumption of the heat pump system, especially the energy efficiency ratio of units, affects the economy and energy saving of the system to a certain extent [6, 7]. The low energy efficiency ratio is mainly due to the high deicing energy consumption of the system, which exceeds the reasonable ice melting heat consumption and also reduces the economy and energy saving of the heat pump system [8].

How to realize the continuous cycle of icing, deicing, ice removal, and refreezing of the system is the key problem for the implementation of the cold- water phase- change energy heat pump system. At present, the existing deicing methods include mechanical scraping, ring-pulling ice scraping, and liquid-solid fluidized bed. The spiral scraper solidification heat exchanger belongs to the mechanical scraper, which relies on a single mechanical force to scrape and remove ice. The motor is connected with the scraper winch through the shaft, and the scraper winch is arranged in the heat exchange tube. The working principle is that the motor drives the scraper winch to rotate in the heat exchange tube, and the scraper scrapes the heat exchange wall. The ice layer on the wall of the heat exchange tube is removed so that the broken ice and water are mixed with cold water. The pull ring type ice cleaning heat exchanger belongs to the single mechanical force outside the tube to deice. The pulley is set at the left and right heads. The pulley is connected to the motor through the lock. The scraper ring is set on the lock and is set outside the heat exchange tube. Its working principle is that the motor drives the scraper ring to move along the heat exchange tube through the lock. The ice layer attached to the heat exchange tube wall is scraped, and the crushed ice under the scraping flows out with cold water. The liquid-solid fluidized bed deicing method relies on the impact of sand and stone on the ice layer of the heat exchanger tube wall, which destroys the ice layer attached to the heat exchanger tube wall to achieve the purpose of deicing [9–11]. The key to the device is how to recycle sand and stone. The device consists of a swirl desander, a regulating valve, and an ejector. The swirl desander and the ejector are connected by a regulating valve. The mixture of sand and ice water flowing out of the heat exchanger enters the cyclone desander. Under the action of centrifugal force, the mixture of sand and ice water is separated, and the sand enters the heat exchanger again with water through the ejector.

Wall icing is a process of continuous growth and expansion after the crystal nucleus is attached to the cold surface [12]. After a long time of operation of the unit, the combination of ice crystals and the wall has been extremely close. In addition, the hardness of the ice layer is large [13]. In order to avoid excessive torque damage to the transmission mechanism, mechanical ice scraping or pulling ring ice scraping needs to start layer by layer from the outermost ice layer, which consumes a lot of electricity and time [14]. Speeding up the deicing speed is prone to hinge tension and blade wear, which makes the heat pump unit have to temporarily shut down and repair, and it greatly reduces the reliability of the unit operation. On the basis of referring to a large number of ice melting and deicing technologies at home and abroad, this study proposes a deicing method combining thermal melting ice and mechanical scraping ice. Firstly, it is heated from the inside of the metal wall to melt the part of the ice layer that is closely contacted with the wall, and then the ice layer is stripped by the scraper. Due to the significant reduction in the adhesion of the ice layer after melting and the buoyancy effect of water, this method can greatly accelerate the deicing speed and reduce the transmission torque and energy consumption. In order to verify the uninterrupted cycle ability of the system for icing, deicing, and refreezing, an experimental platform for the cold-water phase-change energy system was built, and the actual energy consumption characteristics of the system [15] were studied. The relationship between the deicing energy consumption of the system and the effective energy efficiency ratio of the unit and the primary energy utilization rate of the system was further explored, providing a data reference for the subsequent system optimization. This paper mainly analyzes the energy consumption characteristics of the heat pump system from three aspects: energy consumption of deicing, primary energy utilization rate, and unit energy efficiency ratio.

## 2. Experiment of Cold-Water Phase-Change Energy Heat Pump System

### 2.1. Cold-Water Phase-Change Energy Heat Pump System

The principle of the cold-water phase-change energy heat pump system is shown in Figure 1. The system consists of a heat pump unit, a cold-water phase-change machine, an ice-melting heat exchanger, a water tank, a solenoid valve, and a water pump [16]. The water tank and the cold-water phase-change machine are connected by the pipeline to form the ice water cycle, the phase-change heat exchanger and the heat pump unit are connected by the pipeline to form the intermediate water cycle, and the end water cycle is formed between the heat pump unit and the end user. In addition, one end of the plate heat exchanger is connected to the intermediate water outlet pipe, and the other end is connected to the terminal water outlet pipe.

The specific structure of the cold-water phase-change machine is shown in Figure 2 [17–19]. Multiple heat exchange tubes form a heat exchange tube row in the vertical direction. The scraper is fixed on the spindle, and one end of the spindle is connected to the motor. The scraper array is set between the heat exchange tube rows. The working principle is that the cold water enters the cold-water storage tank from the cold-water inlet, and the cold water enters the cold-water channel through multiple cold-water inlets. The cold water is filled with the cold-water channel and heated with the intermediate water below 0°C in the heat exchanger tube. The cold water releases the cold-water phase-change energy and forms ice on the wall surface of the heat exchanger tube. When the ice layer reaches a certain thickness, the electromagnetic valve in the system is opened, and the intermediate water and the end water are heated to enter the heat exchanger tube. The ice layer on the heat exchanger tube wall absorbs heat loss, then the motor starts, the scraper rotates around the spindle, and the loose ice layer is scraped to achieve the effect of completely removing the ice layer from the heat exchanger wall. The ice slurry flows out from the cold-water outlet with the flow.

The cold-water tank heating system consists of four cycles, namely, the cold-water phase-change cycle, the intermediate water cycle, the end cycle, and the intermittent melting cycle [20]. The operation principle of the system is that 0°C cold water in the water tank enters the phase-change energy heat exchanger through the pipeline, and heats with the intermediate water in the phase-change energy heat exchanger. After releasing the phase-change energy, the water is frozen and attached to the heat exchange tube wall. When the ice layer reaches a certain thickness, the deicing cycle is started, and the solenoid valve is opened. The plate heat exchanger leads from the end of the high-temperature hot water to heat the intermediate water. Because the end return water temperature is above 40°C, the intermediate water quickly returns to the temperature. The ice attached to the heat exchanger tube wall absorbs the heat of the intermediate water and falls off the heat exchanger tube wall into the cold-water channel. The scraper of the phase-change energy heat exchanger pulls the ice block up and breaks it, allowing it to flow back to the water tank in the form of an ice-water mixture and complete the cold-water cycle. The intermediate water at −1°C enters the evaporator of the unit, and the heat energy released in the evaporator is reduced to −4°C. The intermediate water at −4°C enters the cold-water phase-change machine and heats the cold water at around 0°C. The absorption phase-change energy rises to −2°C and flows out of the cold-water phase-change machine, thus completing the intermediate water cycle. The end water at 43°C is heated to 50°C by a heat pump to supply users. After users use heat energy, they return to the heat pump unit at 43°C to complete the end cycle.

### 2.2. The Experimental Device and Method

The photo of the experimental device is shown in Figure 3. In the experimental system, the heat pump unit is SRG-650AH, the refrigerant is R22, and the unit runs under 75% load. The inner diameter of the phase-change heat exchange tube is 54 × 19 mm, the outer diameter is 60 × 25 mm, and the total area of heat exchange is 150 m^2^. The total area of the ice melting heat exchanger is 36 m^2^. The intermediate water antifreeze is a 30% glycerol solution and the freezing point is −10°C.

In order to ensure the authenticity and accuracy of the data obtained in this experiment, the winter heating design operation condition used in the cold-water phase-change heat pump system is the actual operation condition of the heat pump system. Under this operating condition, the inlet and outlet temperature of the cold water in the cold-water circulation side of the heat pump system is 0°C/0°C; considering the heat transfer area of the cold-water phase-changer, the inlet and outlet temperature of the intermediate antifreeze on the intermediate circulation side is −1°C/−5°C, and the temperature difference is 4°C; the supply and return water temperature of the end circulation side is 45°C/40°C, and the temperature difference is 5°C.

The main parameters needed to be collected in this experiment are cooling water flow, intermediate water flow, terminal heat supply, deicing heat consumption, inlet and outlet water temperature of the cold-water side of the phase-change heat exchanger, inlet and outlet water temperature of the intermediate water side of the phase-change heat exchanger, inlet and outlet water temperature of the evaporator of the heat pump unit, inlet and outlet water temperature of the condenser of the heat pump unit, unit power consumption, and ice thickness. In order to ensure the accuracy of the experimental data, the data acquisition instrument and the accuracy used in the experiment are shown in Table 1.

In the stage of experimental preparation, according to the operating conditions of the cold-water phase-change energy heat pump system, the operating parameters are set as follows: the freezing time is 80 min; the intermediate water flow is 40 t/h; and the cold-water flow is 75 t/h. In the experiment, when the heat pump unit is turned on, the cold water in the water tank enters the phase-change heat exchanger under the action of the cold-water pump. The cold water on the shell side of the cold-water phase-change machine releases the latent heat of the phase-change to the intermediate water in the tube pass and freezes on the wall of the heat exchange tube. The freezing process is set for 80 minutes. When the freezing time reaches the set value of the system, the heat pump unit is shut down, the ice melting valve is opened for 5 minutes, and the ice discharging motor starts to work. The falling ice layer is discharged into the water tank along with the cold-water channel and discharged by the ice discharge pump. After that, the heat pump unit is turned on and gets heat from freezing, so the cycle goes on and on. After the system runs for two or three cycles, the experimental data is recorded.

### 2.3. Experimental Data Processing

During the operation process of the cold-water phase-change energy heat pump system, the intermediate antifreeze needs to extract part of the heat from the end pipe through the ice melting heat exchanger to melt ice. This part of the energy is called deicing energy consumption, and the ratio between the deicing energy consumption and the unit heating capacity is called the deicing energy consumption proportion. The formula of deicing energy consumption proportion is shown as follows:

(1) $$\begin{array}{c} \varepsilon =\frac{Q_{de}}{Q_{z}}=\frac{Q_{de}}{Q_{de}+Q_{g}}\text{,} \end{array}$$

where *ε* is the deicing energy consumption proportion; *Q*_*de*_ is the deicing energy consumption, kW; *Q*_*z*_ is the unit heating capacity, kW; and *Q*_*g*_ is the terminal heat supply quantity, kW. The heat consumption of deicing and end heating can be measured by ultrasonic heat meter [21].

The COP of heat pump unit under cold-water phase-change condition is as follows:

(2) $$\begin{array}{c} COP=\frac{Q_{z}}{P}\text{,} \end{array}$$

where COP is the coefficient of performance of unit; *P* is the power consumption, kW.

The power consumption can be measured by an electricity meter. The most important index to measure is the energy efficiency ratio of a heat pump unit, which is the ratio of heating capacity *Q* to power consumption *P* [22]. For the cold-water phase-change energy heat pump system, an operation cycle includes the icing process and the deicing process. In every operation cycle, the running condition of the system is constantly changing. The energy efficiency ratio of the heat pump system during operation is calculated by cycle, that is to say, using the data of heating capacity and power consumption in each cycle period.

### 2.4. Error Analysis

Since the experimental results are not directly measured by the experimental instruments, there is the problem of indirect measurement error transmission. The indirect measurement error *y* has the relationship of measurement value *x* shown as follows:

(3) $$\begin{array}{c} y=f\left(x_{1},x_{2}......x_{n}\right)\text{.} \end{array}$$

The maximum absolute error of indirect measurement is as follows:

(4) $$\begin{array}{c} \Delta y=\left|\frac{\partial y}{\partial x_{1}}\right|\Delta x_{1}+\left|\frac{\partial y}{\partial x_{2}}\right|\Delta x_{2}+......+\left|\frac{\partial y}{\partial x_{n}}\right|\Delta x_{n}\text{.} \end{array}$$

According to (1), *Q*_*de*_ is deicing heat consumption and *Q*_*z*_ is unit heating capacity, which is measured by an ultrasonic heat meter, so the absolute error Δ*ε* is calculated as follows:

(5) $$\begin{array}{c} \Delta \varepsilon =\sqrt{\frac{\partial \varepsilon }{\partial Q_{de}}Q_{de}^{2}+\frac{\partial \varepsilon }{\partial Q_{z}}Q_{z}^{2}}\text{.} \end{array}$$

The accuracy level of an ultrasonic heat meter is Level 2, which indicates that the accuracy is between 2% and 3%. If the accuracy is 2%, the error of energy consumption of deicing is 2.8%.

## 3. Results and Discussion

### 3.1. Energy Consumption Analysis of Deicing

During the experiment, the heat consumption of ice melting and the amount of heat supply in each heat exchange cycle are measured by the ultrasonic heat meters set on the ends of the heating pipe, intermediate ice melting return pipe, and terminal ice melting water supply pipe, respectively. The heat consumption of ice melting is the heat loss of the end, and the ratio of heat loss to total heating energy is the proportion of deicing energy consumption.

Figure 4 is the diagram of heat quantity comparison among heat supply at the end, heat consumption of intermediate, and heat consumption at the end of each heat exchange cycle. It can be seen that the heat supply at the end is between 300 kW and 350 kW, and the deicing heat consumption measured is between 37 kW and 47 kW. The experimental data are substituted into (1) to calculate the proportion of deicing energy consumption in each heat exchange cycle.

Figure 5 shows the proportion of deicing energy consumption obtained from the experiment. It is shown that the proportion of deicing energy consumption measured by an intermediate heat meter is always lower than that of terminal energy consumption. This is due to heat loss in the process of heat transfer.

When the end water exchanges heat with intermediate water in the ice melting heat exchanger, part of the heat is transferred to the outside, resulting in heat loss. The measurement error of the two heat meters is within the acceptable range, and the trend chart of the energy consumption ratio obtained from the two experimental data is similar, so it can be judged that the experimental results are reliable. This experiment should be based on the measured data of the heat meter at the end of the ice melting pipe, and the proportion of the deicing energy consumption of the end heat meters of multiple cycles should be counted. The calculation results show that the deicing energy consumption accounts for about 0.135, that is, for every seven units of heat provided by the unit, one unit of heat is used for ice melting.

### 3.2. Analysis of Energy Efficiency Ratio in Unit

In order to ensure the accuracy of the energy efficiency ratio obtained from the experiment and reduce the experimental measurement and calculation error, two different methods are adopted to calculate the unit COP according to the experimental data.

The first method is to calculate the average energy efficiency ratio of each heat exchange cycle indirectly by using a heat meter and an electricity meter based on a heat exchange cycle; the second method is to record the experimental data of each heat exchange cycle and record the real-time change of energy efficiency ratio by using the software provided by the unit, so as to obtain the change of the COP in a heat exchange cycle.

#### 3.2.1. Method I

Since the operation cycle of the cold-water phase-change energy heat pump unit is a heat exchange cycle, the energy efficiency ratio can be obtained by measuring the heating capacity and power consumption of the unit in one heat exchange cycle. In order to ensure the authenticity of the experimental results, a number of groups of experimental data were randomly selected, which are shown in Figures 6 and 7.

The data from Figures 6 and 7 show that the heating capacity of the unit in each heat exchange cycle is maintained between 270 and 330 kW, and the power consumption of the unit is maintained between 80 and 110 kW. The heating capacity and power consumption of the unit are in a fluctuation state within a certain range due to the influence of external temperature and unit states during the operation of the unit. In order to study the change in energy efficiency ratio in the heat pump system during operation, the experimental data of each heat exchange cycle are substituted into (2), the unit energy efficiency ratio of each cycle is calculated, and the energy efficiency ratio of the unit is drawn in Figure 8.

It can be seen from Figure 8 that according to the experimental data of multiple heat exchange cycles, the COP of the heat pump unit is concentrated between 2.8 and 3.5, and the COP of the unit fluctuates slightly within a small range, which is mainly caused by two reasons: (1) it is affected by the error of experimental data recording; and (2) it is affected by the phase converter due to the unstable icing rate. In order to ensure the accuracy of the experimental results, the second method is used to calculate the COP of the unit.

#### 3.2.2. Method II

During the test, a heat exchange cycle is randomly selected, and the real-time COP of the unit is calculated by the software and stored on the computer system. As shown in Figure 9, since the cold-water phase-change energy heat pump unit is in the best state when it starts up, with high evaporation temperature and low condensation temperature, the COP quickly reaches the maximum value from zero.

With the operation of the system, the COP gradually decreases to a certain range and fluctuates steadily until the unit is shut down [23], and the COP is reduced to 0. Considering that the heat pump system operates at a constant flow rate, the unit COP changes as the operation time. The COP of the unit can be expressed by *n*-order polynomial of operation time as follows:

(6) $$\begin{array}{c} f\left(t\right)=p_{1}\cdot x^{n}+p_{2}\cdot x^{n-1}+....+p_{n}\cdot x+p_{n+1}\text{,} \end{array}$$

where *t* is the operating time of unit, min, and *p*_1_, *p*_2_,…, *p*_*n*+1_ are the fit coefficients.

Combined with the correction coefficient given by the heat pump unit manufacturer, the fitting equation of the COP is obtained, and then the average COP of the heat pump system in an operation cycle is obtained.  Figure 10 shows the COP fitting similarity and residual diagram. According to the residual diagram, the quadrinomial residual modulus is 0.67342, the pentanomial residual modulus is 0.59793, and the hexanomic formula residual modulus is 0.57305. The fitting equation of COP is as follows:

(7) $$\begin{array}{c} f\left(t\right)=-1.5\times 10-8t^{5}+3\times 10-6t^{4}-2.3\times 10-4t^{3}+0.00079t^{2}-0.12t+3.8. \end{array}$$

Mean value of integral:

(8) $$\begin{array}{c} f\left(x\right)=\frac{1}{b-a}\int_{a}^{b}f\left(x\right)dx\text{.} \end{array}$$

The average COP is 3.1 calculated by (7), and the COP of the heat pump unit in multiple heat exchange cycles can be calculated by using the same method. So, the COP of the heat pump unit is concentrated between 2.75 and 3.2.

Based on the calculation results of method I and method II, considering that the COP of the unit changes greatly during the start and the end stages of a single heat exchange cycle in the experimental processing, in order to obtain the unit COP during the stable operation of the heat pump system and reduce the experimental error, the intersection of the results of method I and method II is taken, and the COP of the unit is concentrated between 2.8 and 3.2.

For the cold-water phase-change energy heat pump water system, since part of the heat is extracted from the end of the heating pipe to melt ice, the effective COP of the cold-water phase-change energy heat pump unit is as follows:

(9) $$\begin{array}{c} ECOP=\left(1-\varepsilon \right)\cdot COP, \end{array}$$

where ECOP is the effective performance ratio of the unit and *ε*is the proportion of deicing energy consumption.

Substituting the experimental results into (8), the ECOP of the cold-water phase-change energy heat pump unit is 2.42∼2.76.

### 3.3. Energy Consumption Analysis of System

In order to analyze the energy consumption characteristics of the cold-water phase-change energy heat pump system, the primary energy utilization ratios of five heating modes, namely, cold-water phase-change energy heat pump system, sewage source heat pump system [24], ground source heat pump system [25], air source heat pump system [26], and coal-fired boiler coupled water chiller, are compared and analyzed. The primary energy utilization ratio refers to the ratio of the energy obtained to the primary energy consumed [27].

(10) $$\begin{array}{c} PER=\frac{Q_{gain}}{Q_{p}}\text{,} \end{array}$$

where PER is the primary energy utilization rate [28]; *Q*_*p*_ is the primary energy consumption of air conditioning system, kW; and *Q*_gain_ is the primary heat supply of air conditioning system, kW.

The primary energy consumption of coal-fired boiler heating system is *E*_l_.

(11) $$\begin{array}{c} E_{l}=\frac{Q_{r}}{Q_{p}}=\eta_{r}\cdot \eta_{f}\cdot \left(1-\eta_{s}\right)\text{,} \end{array}$$

where *Q*_*r*_ is the energy consumption at the end of heating, kW; *η*_*r*_ is the thermal efficiency of coal fired boiler; *η*_*s*_ is the power transmission efficiency; and *η*_*f*_ is the primary energy generation efficiency.

Then the primary energy utilization ratio of the heat pump system in winter is

(12) $$\begin{array}{c} E_{r}=COP\cdot \eta_{f}\cdot \left(1-\eta_{s}\right)\text{.} \end{array}$$

Taking the winter heating in a certain area of Qingdao as an example, the heating index is 45 W/m^2^ and the total heating time is 120 days. The efficiency of a coal-fired boiler is supposed as 73%; the heating efficiency of a direct-fired unit is supposed as 92%; the COP of an air source heat pump system is 2.7 and that of a ground source heat pump system is 4.5; the COP of a sewage source heat pump system is 4. According to the above experimental data, the COP of the cold-water phase-change energy unit can be taken as 3 [29].

Finally, the primary energy utilization ratio of the cold-water phase-change energy heat pump system is 1.145, the ground source heat pump is 1.354, the sewage source heat pump is 1.290, the air source heat pump is 0.884, and the coal-fired coupling water-cooling unit is 0.901. That is, the primary energy utilization ratio of the cold-water phase-change energy heat pump system is 18.2% lower than the ground source heat pump, 12.7% lower than the sewage water source heat pump, 29.52% higher than the air source heat pump, and 27.08% higher than the coal-fired coupled water-cooling unit.

## 4. Conclusion

In the process of ice discharging, the cold-water phase-change energy heat pump system needs to extract part of the heat from the end heating pipe for ice melting. The deicing energy consumption of the cold-water phase-change energy heat pump system accounts for about 13.5% of the total energy consumption. That is, for every seven units of heat provided by the unit, one unit of heat is used for ice melting. This feature should be fully considered in the system design to meet the continuous operation requirements of the system in order to reduce the energy consumption of deicing.

The COP of the cold-water phase-change energy heat pump unit is about 2.8∼3.2. Considering the deicing energy consumption of the system, the ECOP of the heat pump unit is about 2.42∼2.76. In order to improve the unit energy efficiency ratio [15], the heat pump system should be further optimized to reduce the deicing heat loss and power loss of the system.

The primary energy utilization ratio of the cold-water phase-change energy heat pump system is 1.145, which is 29.52% higher than that of an air source heat pump and also 27.08% higher than that of coal-fired and water-cooled units. Compared with other conventional heating systems, this system has a higher energy utilization ratio, less water demand, better economic and social benefits, and wide engineering application prospects.

## Figures and Tables

**Figure 1:** System schematic of cold-water phase-change energy heat pump.

**Figure 2:** Schematic diagram of cold-water phase-change heat exchanger.

**Figure 3:** Photo of the experimental device.

**Figure 4:** Diagram of heat quantity comparison.

**Figure 5:** Energy consumption ratio of deicing.

**Figure 6:** Heat production of unit.

**Figure 7:** Power consumption of unit.

**Figure 8:** Energy efficiency ratio of unit.

**Figure 9:** Trend of the COP in a cycle.

**Figure 10:** The fitting curves and residuals of COP.

**Table 1:** Measuring instruments.

Name of equipment	Model	Accuracy of measurement
Ultrasonic flowmeter	MIK-2000H	±2%
Ultrasonic heat meter	LDGR-MIK-125	Level 2
Digital thermometer	DTM-402 digital thermometer	±0.2%
Electronic vernier calliper	—	—
Control cabinet data display	—	—
Electric meter	DTSD986	Level 2

## Data Availability

The data used to support the findings of this study are available from the corresponding author upon request.
